# Chronic alcohol exposure exacerbates inflammation and triggers pancreatic acinar-to-ductal metaplasia through PI3K/Akt/IKK

**DOI:** 10.3892/ijmm.2014.2055

**Published:** 2014-12-29

**Authors:** XIN HUANG, XUQI LI, QINGYONG MA, QINHONG XU, WANXING DUAN, JIANJUN LEI, LUN ZHANG, ZHENG WU

**Affiliations:** 1 Department of Hepatobiliary Surgery, First Affiliated Hospital of Xi’an Jiaotong University, Xi’an 710061, P.R. China; 2 Department of General Surgery, Xi’an Central Hospital, Xi’an Jiaotong University, Xi’an 710061, P.R. China; 3 Department of General Surgery, First Affiliated Hospital of Xi’an Jiaotong University, Xi’an 710061, P.R. China

**Keywords:** chronic alcohol, lipopolysaccharide, acinar-to-ductal metaplasia, PI3K/Akt/IKK

## Abstract

Pancreatic acinar-to-ductal metaplasia (ADM) has been identified as an initiating event that can progress to pancreatic intraepithelial neoplasia (PanIN) or pancreatic ductal adenocarcinoma (PDAC). Acini transdifferentiation can be induced by persistent inflammation. Notably, compelling evidence has emerged that chronic alcohol exposure may trigger an inflammatory response of macrophages/monocytes stimulated by endotoxins. In the present study, we aimed to evaluate the role of inflammation induced by chronic alcohol and lipopolysaccharide (LPS) exposure in the progression of pancreatic ADM, as well as to elucidate the possible mechanisms involved. For this purpose, cultured macrophages were exposed to varying doses of alcohol for 1 week prior to stimulation with LPS. Tumor necrosis factor-α (TNF-α) and regulated upon activation, normal T cell expression and secreted (RANTES) expression were upregulated in the intoxicated macrophages with activated nuclear factor-κB (NF-κB). Following treatment with the supernatant of intoxicated macrophages, ADM of primary acinar cells was induced. Furthermore, the expression of TNF-α and RANTES, as well as the phosphatidylinositol-3-kinase (PI3K)/protein kinase B(Akt)/inhibitory κB kinase (IKK) signaling pathway have been proven to be involved in the ADM of acinar cells. Moreover, Sprague-Dawley (SD) rats were employed to further explore the induction of pancreatic ADM by chronic alcohol and LPS exposure *in vivo*. At the end of the treatment period, a number of physiological parameters, such as body weight, liver weight and pancreatic weight were reduced in the exposed rats. Plasma alcohol concentrations and oxidative stress levels in the serum, as well as TNF-α and RANTES expression in monocytes were also induced following chronic alcohol and LPS exposure. In addition, pancreatic ADM was induced through the PI3K/Akt/IKK signaling pathway by the augmented TNF-α and RANTES expression levels in the exposed rats. Overall, we characterized the link between inflammation induced by chronic alcohol and LPS exposure and pancreatic ADM. However, the mechanisms behind the induction of pancreatic ADM warrant further investigation.

## Introduction

A number of studies have clarified that excessive alcohol consumption is the primary etiological factor in the induction of chronic pancreatitis (CP) or even pancreatic cancer (1–3). Both in acute pancreatitis and CP, a high intake of alcohol is an important causative factor; multiple research studies have strived to elucidate the molecular mechanisms responsible for alcohol-induced pancreatic injury (4). In acinar cells, alcohol has been proven to elevate the activation of transcription factors, such as nuclear factor-κB (NF-κB) and cytokine expression (5). Furthermore, alcohol exposure can induce an increase in cytoplasmic calcium ions (Ca^2+^) levels, which leads to mitochondrial depolarization and necrosis (6).

The association between alcoholic pancreatitis and susceptibility factors, including genetic polymorphisms (7), minor cystic fibrosis mutations (8) and environmental factors, such as bacterial endotoxins have been examined (9). Plasma endotoxin levels have been shown to be higher in drinkers than in non-drinkers and are known to correlate with the severity of alcoholic liver disease (10). Notably, an increase in gut permeability may be induced by alcoholic intoxication, which allows gut bacteria or bacterial products to enter the portal circulation (11). Notably, a positive correlation has been demonstrated between higher circulating lipopolysaccharide (LPS) levels and an increased severity of acute pancreatitis (12).

Alcohol consumption may lead to the enhanced production of pro-inflammatory cytokines and chemokines. Alcoholic hepatitis and pancreatitis, two major clinical complications of chronic alcohol use, have been shown to be intimately associated with increasing circulating levels of pro-inflammatory cytokines that predict poor clinical outcomes (13,14). Previous studies have indicated that acute alcohol can inhibit pro-inflammatory cell activation, which is pivotal to innate immune activation (15). By contrast, chronic alcohol exposure leads to the elevated activation of pro-inflammatory cytokines in humans (16). Human monocytes, following treatment with prolonged alcohol *in vitro*, have been shown to produce increased levels of tumor necrosis factor-α (TNF-α) and have shown elevated NF-κB activation (17). Additionally, chronic alcohol intake may persistently activate monocytes and macrophages, resulting in a marked increase in the levels of in pro-inflammatory cytokines, such as TNF-α, interleukin-1 (IL-1) and interleukin-1 (IL-6) and the chemokine interleukin-8 (IL-8) (18–20).

Chronic inflammation may cause cellular transdifferentiation which can occur in a number of organs, including the pancreas (21), stomach (22), intestine (23) and esophagus (24). Pancreatic acinar-to-ductal metaplasia (ADM) has been identified as an initiating event that can trigger the development of serious lesions, such as pancreatic intraepithelial neoplasia (PanIN) or pancreatic ductal adenocarcinoma (PDAC) (21,25). ADM, as a reversible process, can be induced by activating K-ras mutations, epidermal growth factor receptors or pancreatic inflammation (26–28). A previous study on patients with duct-like metaplasia induced by CP demonstrated a 16-fold increase in the relative risk for PDAC, increasing to 50-fold in patients with familial CP (29).

In the pancreas, chronic alcohol exposure has been reported to exacerbate the degree of fibrosis induced by LPS through an augmented level of tumor growth factor-β (TGF-β) (30). However, it remains largely unknown whether the inflammation induced by chronic alcohol and LPS may contribute to pancreatic ADM. In the present study, we aimed to evaluate the role of inflammation induced by chronic alcohol and LPS exposure in the progression of pancreatic ADM, as well as to elucidaste the possible mechanisms involved. For this purpose, cultured macrophages were exposed to varying doses of alcohol for 1 week prior to LPS stimulation. TNF-α regulated upon activation, normal T cell expression and secreted (RANTES) expression was upregulated in the intoxicated macrophages with activated NF-κB. Following treatment with the supernatant of intoxicated macrophages, ADM of primary acinar cells was induced. Furthermore, TNF-α and RANTES expression, as well as the phosphatidylinositol-3-kinase (PI3K)/protein kinase B (Akt)/inhibitory κB kinase(IKK) signaling pathway, have been shown to be involved in the ADM of acinar cells. Moreover, Sprague-Dawley (SD) rats were employed to explore the induction of pancreatic ADM by chronic alcohol and LPS exposure. Some physiological parameters, such as body weight, liver weight (LW) and pancreatic weight (PW) were reduced in the exposed rats. Plasma alcohol concentrations and oxidative stress levels in the serum along with TNF-α and RANTES expression levels in monocytes were also induced following chronic alcohol and LPS exposure. In addition, pancreatic ADM was induced through the PI3K/Akt/IKK signaling pathway by augmented TNF-α and RANTES levels in the exposed rats.

## Materials and methods

### Alcohol exposure and stimulation of cells

A rat macrophage cell line obtained from ScienCell Research Laboratories (Carlsbad, CA, USA) was cultured in macrophage medium (MaM, Cat. no. 1921) according to the manufacturer’s instructions. The macrophages were stimulated with varying doses (0, 5, 10, 15, 20 and 25 mM) of alcohol [ethanol (EtOH)] for 1 week prior to treatment with *Escherichia coli*-derived LPS (100 ng/ml). The ethanol concentration was selected according to a previous study (33). Ethanol (25 mM) *in vitro* is approximately equal to a blood alcohol level of 0.1 g/dl, which is achieved *in vivo* after a dose of moderate alcohol. Cell viability was not affected by ethanol or LPS treatment (data not shown).

### Isolation of primary pancreatic acinar cells

The isolation of primary pancreatic acinar cells was as previously described (31). Briefly, the pancreas was removed, washed twice with ice-cold PBS, minced into 1–5-mm sections and digested with collagenase I (37°C with a shaker). The collagen digestion was terminated by the addition of an equal volume of ice-cold PBS. The digested pancreatic sections were washed twice with PBS containing 5% FBS and pipetted through a 500-*μ*m mesh and then a 105-*μ*m mesh. The supernatant of this cell suspension containing acinar cells was added dropwise to 20 ml PBS containing 30% FBS. The acinar cells were then pelleted (1,000 rpm for 2 min at 4°C) and resuspended in 10 ml Waymouth complete medium (1% FBS, 0.1 mg/ml trypsin inhibitor and 1 *μ*g/ml dexamethasone).

### Animals and treatment

A total of 120 8-week old male SD rats were purchased from Shanghai SLAC Laboratory Animal Co., Ltd. (Shanghai, China). The animals were housed under standard conditions with a 12/12-h light/dark cycle at room temperature and fed a common diet with free access to water. To establish chronic alcoholic and LPS-stimulated rat models, the SD rats were randomly divided into 6 groups and intraperitoneally injected with 0, 5, 10, 15, 20 and 25 mmol/kg/day alcohol [ethanol (EtOH)] for 4 weeks. Following alcohol exposure, a dose (1 mg/kg) of LPS was administered by intravenous injection. For TNF-α and RANTES neutralization, the rats were injected with anti-TNF-α (sc-8301; Santa Cruz Biotechnology, Santa Cruz, CA, USA) or anti-RANTES (sc-514019; Santa Cruz Biotechnology) antibodies. The doses of anti-TNF-α or anti-RANTES antibody w as based on the results of preliminary experiments. To inhibit PI3K or IKK activity in rats, LY294002 (a PI3K inhibitor; 100 mg/kg, 10 min before the alcohol injection) was intravenously injected; 25% dimethyl sulfoxide in PBS was used as the vehicle.

All animal experimental procedures were conducted under the guidelines of the National Health and Medical Research Council for the Care and Use of Animals for Experimental Purposes in China. All efforts were made to minimize the suffering of the animals.

### siRNA transfection

Scrambled siRNA and small-interfering RNA (siRNA) targeting NF-κB or the IL-1 receptor-associated kinase (IRAK)-M was purchased from Santa Cruz Biotechnology. The cells were transfected with scrambled or NF-κB/IRAK-M siRNA according to the manufacturer’s instructions. Briefly, the NF-κB/IRAK-M and scrambled siRNA (30 pmol) were diluted in 500 *μ*l DMEM and mixed with 5 *μ*l Lipofectamine RNAiMAX (Invitrogen, Carlsbad, CA, USA). Following 15 min of incubation at room temperature, the complexes were added to the cells to a final volume of 3 ml medium. The cells were then harvested at the indicated times for further analysis. The efficiency of the NF-κB/RAK-M siRNA was confirmed by western blot analysis of Flag expression.

### Adenovirus construction

All recombinant adenoviruses were constructed according to a previous report (32). Briefly, IκB or IRAK-M were amplified and subcloned into pAdTrack-CMV, an adenoviral shuttle plasmid, whereas GFP was used as a non-specific control. Subsequently, the recombinant shuttle plasmids, pAdTrack-CMV and pAdEasy-1, were homologously recombined in the *Escherichia coli* strain BJ5183. The recombinant plasmids obtained were transfected into HEK293 cells to generate recombinant adenovirus. The virus was amplified and purified, and titers were determined using the p24 ELISA kit (Cell Biolabs, Inc., San Diego, CA, USA), before being stored at −80°C for subsequent use.

### Reporter gene assays

The acinar cells were infected with adenovirus-NF-κB-luciferase adenovirus (at 10^7^ IFU/ml), and immediately plated on a 24-well plate and cultured with 6 groups of macrophage supernatants. At 24 and 48 h after infection, the cells were collected and washed with ice-cold PBS, lysed using 250 *μ*l Passive Lysis Buffer (Promega, Madison, WI, USA) and centrifuged (13,000 rpm for 10 min at 4°C). Assays for luciferase activity were performed according to the luciferase assay protocol (Promega) and measured using a luminometer (Veritas; Symantec) and GloMax software (Promega).

### Detection of plasma alcohol, malondialdehyde (MDA)a nd glutathione peroxidase (GPx) levels, and superoxide dismutase (SOD) activity

A Biochemical Analysis kit (Nanjing Jiancheng Bioengineering Institute, Nanjing, China) was used to measure the plasma alcohol concentration, MDA content, GPx and SOD activity according to the manufacturer’s instructions. Each experiment was performed no less than 3 times.

### Enzyme-linked immunosorbent assay (ELISA) for TNF-α and RANTES detection

The levels of TNF-α and RANTES in the serum were analyzed using a commercially available ELISA kit (Yanjin Biotechnology Co., Shanghai, China) according to the manufacturer’s instructions. The absorbance was read at 450 nm using a 680XR microplate reader (Bio-Rad Laboratories, Hercules, CA, USA). All the samples were analyzed in duplicate. The standard curve for the estimation of TNF-α and RANTES expression was created by linear regression analysis.

### RNA extraction and quantitative reverse transcription-polymerase chain reaction (RT-qPCR)

RNA was extracted from the macrophages or acinar cells using TRIzol RNA extraction reagent (Gibco, Rockville, MD, USA) according to the manufacturer’s instructions. Approximately 5 *μ*g total RNA for each sample were reverse transcribed into first strand cDNA for RT-qPCR analysis. RT-qPCR was performed in a final volume of 10 *μ*l, which contained 5 *μ*l of SsoFast™ EvaGreen Supermix (Bio-Rad Laboratories), 1 *μ*l of cDNA (1:50 dilution) and 2 *μ*l each of the forward and reverse primers (1 mM). The steps used for RT-qPCR were as follows: 94°C for 2 min for initial denaturation; 94°C for 20 sec, 58°C for 15 sec, and 72°C for 15 sec; 2 sec for plate reading for 40 cycles; and a melt curve from 65 to 95°C. β-actin was used as a quantitative and qualitative control to normalize gene expression. Data were analyzed using the formula: R = 2-^(ΔCt sample − ΔCt control)^. The sequences of all the primers used in this experiment are presented in Table I.

### Western blot analysis

The cells were homogenized and lysed with RIPA lysis buffer (100 mM NaCl, 50 mM Tris-HCl pH 7.5, 1% Triton X-100, 1 mM EDTA, 10 mM β-glycerophosphate, 2 mM sodium vanadate and protease inhibitor). Protein concentration was assayed using a Micro BCA Protein kit (Pierce, Rockford, IL, USA). Forty micrograms of protein per lane were separated by 12% SDS-PAGE and electroblotted onto nitrocellulose membranes (Amersham Pharmacia, Munich, Germany). Subsequently, non-specific binding was blocked by incubating with 5% non-fat milk in TBST buffer at room temperature for 1 h. Immunodetection of target proteins [TNF-α, RANTES, IκB, phosphorylated (p-)Akt, p-p38 mitogen-activated protein kinase (MAPK), p-c-Jun amino-terminal kinase (JNK), amylase, cytokeratin-19 (CK-19), total caspase-3, cleavage caspase-3 and β-actin] was performed using mouse monoclonal antibody (1:1,000; Santa Cruz Biotechnology) and anti-β-actin antibody (Sigma, St. Louis, MO, USA), respectively. Goat anti-mouse IgG (1:5,000; Sigma) followed by enhanced chemiluminescence (ECL, Amersham Pharmacia, Piscataway, NJ, USA) was used for detection. BandScan 5.0 software was used for the quantification of all the proteins after western blot analysis.

### Immunohistochemical analysis of amylase and CK-19

A sequential method for amylase/CK-19 double staining was used according to the immunohistochemistry enzyme double staining protocol described in a previous study (34). Briefly, the sections were incubated with goat polyclonal anti-CK19 antibody (dilution 1:100; Santa Cruz Biotechnology) as the first primary antibody and detected using the DAB substrate chromogen system (Sigma). The sections were then blocked again with normal serum, and incubated with the second primary antibody, mouse monoclonal anti-amylase antibody (dilution 1:100; Santa Cruz Biotechnology), after incubating with the anti-mouse secondary antibody and avidin-biotin-peroxidase complex; 3-amino-9-ethylcarbazole (AEC) peroxidase substrate with a characteristic red color was used to detect positive staining and to distinguish from the brown color of DAB. The negative control was established by replacement of the primary antibody with normal serum. Specific antibody-labeled signals were analyzed under a microscope (Nikon, Tokyo, Japan).

### Statistical analysis

Data are expressed as the means ± SD. Statistical significance was analyzed with the one-way factorial ANOVA or the Student’s two-tailed t-test. A value of P<0.05 was considered to indicate a statistically significant difference. All analyses were conducted using SPSS software (SPSS, Inc., Chicago, IL, USA).

## Results

### TNF-α and RANTES expression induced by LPS is enhanced by chronic alcohol exposure

To explore the effects of chronic alcohol on TNF-α and RANTES expression induced by LPS, we cultured rat macrophages (Fig. 1A) with varying doses (0, 5, 10, 15, 20 and 25 mM) of alcohol for 1 week and then treated them with LPS for 1 h. At the end of the treatment, the expression levels of TNF-α and RANTES in these cells were detected by RT-qPCR. The results revealed that the expression levels of TNF-α and RANTES were continuously elevated by alcohol exposure in a dose-dependent manner (Fig. 1B). This was further confirmed by western blot analysis. NF-κB activity was proven to be essential for TNF-α and RANTES expression (Fig. 1C and D). Therein, the expression of IκB, as an inhibitory protein for NF-κB, was analyzed by western blot analysis. Compared to the control group (0 mM alcohol), chronic alcohol exposure clearly reduced the level of IκB expression, implying NF-κB activation (Fig. 1E and F).

### Knockdown of NF-κB/overexpression of IκB lead to the reduction of TNF-α and RANTES expression induced by LPS and chronic alcohol exposure

To further confirm the role of NF-κB and IκB in the regulation of TNF-α and RANTES expression, cultured rat macrophages were transfected with siRNA targeting NF-κB or adenovirus encoding IκB. These cells were then exposed to alcohol (0 or 25 mM) and LPS (100 ng/ml) as depicted above. The expression of TNF-α and RANTES was analyzed by RT-qPCR. The knockdown of NF-κB or the overexpression of IκB significantly decreased the expression of TNF-α and RANTES (Fig. 2).

### The IRAK-M/p38 MAPK/JNK signaling pathway mediates the regulation of TNF-α and RANTES expression

It has been well established that IRAK-M plays a vital role in activating NF-κB and in the regulation of inflammation induced by alcohol and LPS (35,36). Rat macrophages were cultured in the presence of varying doses (0, 5, 10, 15, 20 and 25 mM) of alcohol for 1 week prior to LPS stimulation. IRAK-M expression was analyzed in the exposed macrophages by western blot analysis. As shown in Fig. 3, chronic alcohol markedly impeded IRAK-M expression (Fig. 3A and B). Moreover, the expression of p-p38 MAPK and p-JNK was also examined by western blot analysis. The expression levels of p-p38 MAPK and p-JNK were upregulated by chronic alcohol and LPS exposure (Fig. 3C and D). Furthermore, to explore the role of IRAK-M in the regulation of TNF-α and RANTES expression, we further transfected siRNA targeting IRAK-M into the rat macrophages. The knockdown of IRAK-M induced an increase in p-p38 MAPK and p-JNK expression, as well as TNF-α and RANTES expression in these cells (Fig. 3E and F).

### ADM is induced by culture supernatants of rat macrophages

Liou *et al* (31) proved that macrophages induce ADM in a co-cultured context. In the present study, we hypothesized that chronic alcohol promotes the activation of macrophages induced by LPS and, thus, leads to ADM. To validate this hypothesis, rat macrophages were cultured in the presence of varying doses (0, 5, 10, 15, 20 and 25 mM) of alcohol. Following culture for 1 week, 6 groups of cells were stimulated with LPS prior to collection of the supernatant. Primary acinar cells were isolated from 30 rats and then cultured with macrophage conditioned medium (collected supernatant). In order to detect ADM, the expression of amylase for acinar markers and CK-19 for ductal markers was analyzed by western blot analysis. Compared to the controls (untreated cells), the conditioned medium derived from alcohol- and LPS-treated macrophages showed markedly decreased amylase expression and increased CK-19 expression (Fig. 4A and B).

The progression of ADM has been shown to be implicated in a process of transdifferentiation and the induction of anti-apoptosis (21,37). In the present study, sought to analyze the expression of caspase-3 in acinar cells exposed to macrophage-conditioned medium. As can be seen from the results of western blot analysis, the cleavage of caspase-3 in the acinar cells was evidently downregulated (Fig. 4C and D).

To further investigate the effects of TNF-α and RANTES on ADM, we employed neutralizing antibodies (NABs) to antagonize TNF-α and RANTES. As a result, neutralizing TNF-α and RANTES markedly reversed the effects on amylase and CK-19 expression (Fig. 4E and F).

### The PI3K/Akt/IKK signaling pathway plays a vital role in NF-κB activation induced by rat macrophage supernatants

NF-κB activation and translocation into the nucleus has been proven to be an essential process for initiating ADM (31). In this study, to examine NF-κB activation, we introduced an NF-κB-luciferase reporter into the acinar cells via an adenoviral transduction system. The results revealed that treatment with macrophage supernatants markedly promoted the activity of NF-κB (Fig. 5A). Importantly, compelling evidence has indicated that the PI3K/Akt/IKK signaling pathway may be involved in the activation of NF-κB (38,39). In the present study, PI3K inhibitor LY294002 (25 mM) was added to the cultured primary acinar cells prior to treatment with macrophage supernatants. The expression of the phosphorylated form of Akt and IKK was then analyzed by western blot analysis. Compared to the controls (vehicle-treated group), the inhibition of PI3K led to a decrease in phosphorylated Akt and IKK expression (Fig. 5B). Furthermore, NF-κB activity in the acinar cells was also detected. The results revealed that PI3K inhibition markedly abated NF-κB activity in the acinar cells (Fig. 5C and D).

### Physiological parameters of exposed rats

To explore the effects of chronic alcohol and LPS on the physiological parameters of rats, the animals were injected with a series of doses (0, 5, 10, 15, 20 and 25 mmol/kg/day) of alcohol for 4 weeks and then LPS (1 mg/kg). Following the completion of treatment, all the animals were weighed and then sacrificed by cervical dislocation, with their organs harvested for the calculation of PW, LW, spleen weight (SW) and kidney weight (KW). Compared to the control group (no treatment), increasing the dose of alcohol significantly decreased BW, PW and LW in the rats (Table II). However, no difference was observed in the SW and KW of these rats among all groups (Table II).

To determine the plasma alcohol concentration in the rats, blood samples of these exposed rats were collected and detected by enzyme-based assays. The plasma alcohol concentrations of the exposed rats were much higher than those of the controls. The results revealed that chronic alcohol exposure induced an increase in the plasma alcohol concentration in the rats (Fig. 6A).

To determine oxidative stress caused by chronic alcohol and LPS exposure, the MDA level, SOD activity and GPx activity were calculated with the blood samples collected. Exposure to chronic alcohol and LPS induced an increase in the MDA level in serum with a concurrent decrease in SOD and GPx activity (Fig. 6B–D).

### The levels of TNF-α and RANTES expression in serum and monocytes are increased in rats

To investigate the effects of chronic alcohol and LPS on circulating TNF-α and RANTES expression, TNF-α and RANTES expression in serum was analyzed by ELISA. The results revealed that the levels of TNF-α and RANTES in serum were evidently increased by chronic alcohol and LPS exposure (Fig. 7A). Furthermore, monocytes in blood samples were separated prior to TNF-α and RANTES expression in these cells and were analyzed by RT-qPCR. Compared to the controls, the expression levels of TNF-α and RANTES were distinctly upregulated by chronic alcohol and LPS exposure (Fig. 7B).

### ADM is observed in pancreatic acinar cells of rats

To further determine whether ADM occurs in pancreatic acinar cells of rats exposed to chronic alcohol and LPS, acinar cells derived from the exposed rats were isolated. Amylase and CK-19 expression in these cells were analyzed by western blot analysis. Chronic alcohol and LPS exposure significantly downregulated amylase expression, but enhanced CK-19 expression in the acinar cells compared with the controls (Fig. 8A and B).

We then explored whether ADM is inhibited as TNF-α and RANTES is antagonized *in vivo*. Prior treatments with NABs for neutralizing TNF-α and RANTES were carried out prior to alcohol exposure (0, 25 mmol/kg/day)/LPS (1 mg/kg) in the rats. At the end of treatment, these rats were then sacrificed and the pancreases were harvested for the isolation of acinar cells. Amylase and CK-19 expression in these cells was analyzed by western blot analysis. Compared with the controls, neutralizing TNF-α and RANTES induced an increase in amylase and a decrease in CK-19 expression in at the translational level (Fig. 8C and D).

### The PI3K/Akt/IKK pathway plays an essential role in the induction of pancreatic ADM in vivo

To further examine the role of the PI3K/Akt/IKK pathway in the induction of pancreatic ADM *in vivo*, the animals were administered PI3K inhibitor (LY294002, 100 mg/kg) 10 min piror to exposure to chronic alcohol (0 and 25 mmol/kg/day) and LPS (1 mg/kg). As soon as the treatments were completed, these animals were sacrificed and their pancreases were fixed in formalin. Pancreatic sections were immunostained for amylase and CK-19. As illustrated in the Fig. 8E, the inhibition of PI3K was sufficient to block pancreatic ADM in the rats.

## Discussion

Several studies have indicated that inflammation of the pancreas may be an important source for the initiation of pancreatic cancer (40–42). Reprogramming of pancreatic acini has been shown to occur under many contexts and contributes to acini transdifferentiation (43). It has been demonstrated that chronic alcohol exposure elevates the sensitivity of macrophages/monocytes and boosts the inflammatory response to LPS stimulation (33). The role of alcohol and LPS intoxication in the pancreas and the induction of pancreatic lesions, and eventually, pancreatic cancer remains largely unknown. In the present study, we provide evidence of the mechanisms through which chronic alcohol modulates macrophage/monocyte responses and causes acini transdifferentiation in the pancreas.

It is well established that acute alcoholic exposure inactivates monocyte/macrophage responses to LPS stimulation, while chronic exposure has the opposite effect (33,44). In this study, we found that prolonged exposure to varying doses of alcohol resulted in an increased expression of TNF-α and RANTES in rat macrophages stimulated with LPS. The expression and secretion of pro-inflammatory cytokines in macrophages have been proven to correlate with the enhanced activity of NF-κB (45). In the present study, an increased activity of NF-κB was observed in the macrophages treated with alchohol and LPS with the upregulated expression of cytokines. However, when NF-κB activity was hindered by the knockdown of NF-κB expression or the overexpression of IκB, the expression of TNF-α and RANTES in the macrophages was evidently downregulated.

IRAK-M is one of the primary targets in macrophages exposed to alcohol (46). The decreased expression of IRAK-M was induced in our study in intoxicated macrophages. IRAK-M, as an upstream participant of several pathways, regulates a cluster of factors which include MAPKs and JNK and eventually activates NF-κB (47). In the present study, we found that abated IRAK-M led to the increased expression of p38 MAPK and JNK, as well as the secretion of TNF-α and RANTES. By contrast, the increased IRAK-M expression evidently decreased TNF-κ and RANTES secretion induced by prolonged exposure to alcohol and LPS stimulation. These results indicate that IRAK-M, p38 MAPK and JNK play an important role in the expression of pro-inflammatory cytokines in macrophages exposed to chronic alcohol and LPS.

The transdifferentiation of acinar cells to duct-like cells may lead to metaplastic duct lesions which are commonly observed in pancreatitis (48). In the present study, culture supernatants of intoxicated macrophages contributed to the process of ADM in primary acinar cells. Furthermore, neutralizing TNF-α and RANTES in the supernatant by NABs significantly abolished ADM in the pancreatic acini. These results suggest the role of TNF-α and RANTES in the induction of ADM, which is consistent with the results of the study by Liou *et al* (31).

PI3K activation has been implicated in the pathogenesis of various pancreatic lesions (49). The PI3K/Akt signaling pathway mediates cell proliferation and invasiveness in pancreatic cancer cells. The inhibition of PI3K signaling has been shown to lead to abruption in G1-to-S phase progression and proliferation in pancreatic cancer cells (50). In this study, we found that the inhibition of PI3K resulted in a decrease in pAkt/IKK expression and NF-κB activity induced by macrophage culture supernatant. Given that NF-κB activity dominates ADM in acinar cells, our data demonstrated that the PI3K/Akt/IKK pathway was intimately associated with pancreatic ADM.

Evidence has indicated that a dedifferentiation process may be a crucial part in ADM. Cultured pancreatic acini will undergo apoptosis under normal conditions. However, once pancreatic ADM has been induced, acinar cells can attain a longer lifespan and proliferative properties (51). In the present study, treatment with cultured supernatants of stimulated macrophages induced a downregulation of the expression of cleaved caspase-3 in acinar cells. Thus, an anti-apoptotic process may be induced in acinar cells by the administration of macrophage culture supernatants.

Our results demonstrated that chronic alcohol exposure and LPS stimulation may have an adverse effect on rats. The body weight, PW and LW of the intoxicated rats were significantly reduced at the end of treatment. Moreover, the injection of alcohol and LPS enhanced the level of alcohol and oxidative stress in the serum. Serum TNF-α and RANTES levels examined by ELISA were distinctly augmented in the exposed rats compared with the controls. Additionally, we found that TNF-α and RANTES expression in monocytes in peripheral blood were evidently upregulated by chronic alcohol exposure.

The monocyte secretion of cytokines, such as TNF-α or RANTES plays a central role in the pathophysiology of pancreatitis (52). In this study, we detected the increased expression of CK-19 and decreased amylase expression in acinar cells derived from alcoholic rats, which indicated the occurrence of ADM induced by chronic alcohol and LPS exposure. By contrast, neutralizing TNF-α and RANTES by antibodies led to a decrease in pancreatic ADM. These data provide evidence that TNF-α and RANTES play a major role in the induction of ADM.

We observed that the PI3K/Akt/IKK pathway mediated ADM induction by macrophage supernatants in cultured primary acini. Accordingly, the inhibition of PI3K or IKK in the acini of rats also significantly blocked ADM progression, which suggests the role of PI3K/Akt/IKK in the induction of ADM *in vivo*.

Collectively, we found that chronic alcohol exposure may promote cytokine secretion in macrophages/monocytes stimulated by LPS both *in vitro* and *in vivo*. Under the conditions of higher levels of pro-inflammatory cytokines, pancreatic acini may undergo transdifferentiation which can be blocked by PI3K or IKK inhibition. Since ADM is prevalent in pancreatitis and can progress to advanced cancerous lesions, targeting the PI3K/Akt/IKK pathway may be a promising approach for the treatment of pancreatic ADM.

## Figures and Tables

**Figure 1:** Chronic alcohol exposure upregulates tumor necrosis factor (TNF)-α and regulated upon activation, normal T cell expression and secreted (RANTES) expression in rat macrophages. (A) Cultured rat macrophages (magnification, ×400, F200). (B) mRNA expression of TNF-α and RANTES in rat macrophages exposed to varying doses (0, 5, 10, 15, 20 and 25 mM) of alcohol [ethanol (EtOH)] and lipopolysaccharide (LPS); ^*^P<0.05 vs. 0 mM EtOH + LPS group. (C) Protein expression of TNF-α and RANTES in rat macrophages exposed to varying doses (0, 5, 10, 15, 20 and 25 mM) of alcohol and LPS. (D) Protein expression was analyzed using BandScan 5.0 software and normalized to β-actin; ^*^P<0.05 vs. 0 mM EtOH + LPS. (E) Western blot analysis of IκB expression in rat macrophages exposed to varying doses (0, 5, 10, 15, 20 and 25 mM) of alcohol and LPS. (F) Protein expression was analyzed using BandScan 5.0 software and normalized to β-actin; ^*^P<0.05 vs. 0 mM EtOH + LPS.

**Figure 2:** Nuclear factor (NF)-κB is involved in the regulation of tumor necrosis factor (TNF)-α and regulated upon activation, normal T cell expression and secreted (RANTES) expression in rat macrophages. (A) NF-κB expression was targeted by specific siRNA in macrophages prior to exposure to 25 mM alcohol [ethanol (EtOH)] and LPS. ^*^P<0.05 vs. control, ^**^P<0.05 vs. EtOH + LPS group; (B) IκB (inhibitor NF-κB) of overexpression was induced following transfection with adenovirus into macrophages prior to exposure to 25 mM alcohol and LPS. ^*^P<0.05 vs. control, ^**^P<0.05 vs. EtOH + LPS group.

**Figure 3:** Interleukin-1 receptor-associated kinase (IRAK)-M/p38 mitogen-activated protein kinase (MAPK)/c-Jun amino-terminal kinase (JNK) plays a vital role in the regulation of tumor necrosis factor (TNF)-α and regulated upon activation, normal T cell expression and secreted (RANTES) expression in rat macrophages. (A) Protein expression of IRAK-M in rat macrophages exposed to varying doses (0, 5, 10, 15, 20 and 25 mM) of alcohol [ethanol (EtOH)] and lipopolysaccharide (LPS). (B) Protein expression was analyzed using BandScan 5.0 software and normalized to β-actin; ^*^P<0.05 vs. 0 mM EtOH + LPS. (C) Expression of phosphorylated (p-)p38 MAPK and p-JNK was enhanced in rat macrophages exposed to varying doses (0, 5, 10, 15, 20 and 25 mM) of alcohol and LPS. (D) Protein expression was analyzed using BandScan 5.0 software and normalized to β-actin; ^*^P<0.05 vs. 0 mM EtOH + LPS group. (E) IRAK-M expression was targeted by specific siRNA in macrophages prior to exposure to 25 mM alcohol and LPS. Protein expression of p-p38 MAPK, p-JNK, TNF-α and RANTES was analyzed by western blot analysis. (F) Protein expression was analyzed using BandScan 5.0 software and normalized to β-actin, ^*^P<0.05 vs. control; ^**^P<0.05 vs. 25 mM EtOH + LPS group.

**Figure 4:** Amylase and cytokeratin-19 (CK-19) expression is altered in acinar cells cultured with macrophage supernatant. (A) Rat macrophages were exposed to varying doses (0, 5, 10, 15, 20 and 25 mM) of alcohol [ethanol (EtOH)]. After exposure for 7 days, lipopolysaccharide (LPS; 100 ng/ml) was added. Supernatants of each group were harvested and added into isolated primary acinar cells. Following culture for 48 h, the protein expression of amylase and cytokeratin-19 (CK-19) in acinar cells was analyzed by western blot analysis. (B) Protein expression was analyzed using BandScan 5.0 software and normalized to β-actin; ^*^P<0.05 vs. 0 mM macrophage supernatant. (C) Expression of total caspase-3 and cleaved caspase-3 in acinar cells was analyzed by western blot analysis. (D) Protein expression was analyzed using BandScan 5.0 software and normalized to β-actin; ^*^P<0.05 vs. 0 mM macrophage supernatant. (E) Tumor necrosis factor (TNF)-α and regulated upon activation, normal T cell expression and secreted (RANTES) expression in supernatant was neutralized by anti-TNF-α and anti-RANTES antibodies before the macrophage supernatants were added into the cultured acinar cells. Following treatment for 48 h, the expression of amylase and CK-19 in acinar cells was analyzed by western blot analysis. (F) Protein expression was analyzed using BandScan 5.0 software and normalized to β-actin; ^*^P<0.05 vs. control, ^**^P<0.05 vs. macrophage supernatant group.

**Figure 5:** The phosphatidylinositol-3-kinase (PI3K)/protein kinase B (Akt)/inhibitory κB kinase(IKK) signaling pathway is involved in nuclear factor (NF)-κB activation induced by macrophage supernatant. (A) NF-κB activity was augmented by macrophage supernatant, ^*^P<0.05 vs. control. (B) p-Akt and p-IKK were reduced by LY294002 (PI3K inhibitor). (C) Protein expression was analyzed using BandScan 5.0 software and normalized to β-actin; ^*^P<0.05 vs. macrophage supernatant group. (D) NF-κB activity was reduced by LY294002; ^*^P<0.05 vs. macrophage supernatant group.

**Figure 6:** Variation of plasma alcohol and oxidative stress in rats is caused by chronic alcohol and lipopolysaccharide (LPS) exposure. (A) Plasma alcohol was increased in rats exposed to alcohol [ethanol (EtOH)] and LPS; ^*^P<0.05 vs. control (0 mM/kg/day). (B) MDA levels were elevated in rats exposed to alcohol and LPS; ^*^P<0.05 vs. control (0 mM/kg/day). (C) GPx activity was reduced in rats exposed to alcohol and LPS; ^*^P<0.05 vs. control (0 mM/kg/day). (D) SOD activity was reduced in rats exposed to alcohol and LPS, ^*^P<0.05 vs. control (0 mM/kg/day).

**Figure 7:** Increased expression of tumor necrosis factor (TNF)-α and regulated upon activation, normal T cell expression and secreted (RANTES) is induced by chronic alcohol [ethanol (EtOH)] and lipopolysaccharide (LPS) exposure. (A) Circulating TNF-α and RANTES levels were promoted in rats exposed to alcohol and LPS; ^*^P<0.05 vs. control (0 mM/kg/day). (B) The expression of TNF-α and RANTES was promoted in monocytes of rats exposed to alcohol and LPS; ^*^P<0.05 vs. control (0 mM/kg/day).

**Figure 8:** Pancreatic acinar-to-ductal metaplasia (ADM) was induced in rats by chronic alcohol [ethanol (EtOH)] and lipopolysaccharide (LPS) exposure. (A) Amylase expression was downregulated in pancreatic acinar cells with an enhancement in cytokeratin-19 (CK-19) expression. (B) Protein expression was analyzed using BandScan 5.0 software and normalized to β-actin; ^*^P<0.05 vs. control (0 mM/kg/day). (C) Restoration of amylase expression was caused by neutralizing antibodies with the decreased expression of CK-19. (D) Protein expression was analyzed using BandScan 5.0 software and normalized to β-actin; ^*^P<0.05 vs. control, ^**^P<0.05 vs. EtOH + LPS group. (E) CK-19 and amylase expression in pancreatic sections was detected by immunohistology. Pancreatic ADM was blocked by LY294002 [phosphatidylinositol-3-kinase (PI3K) inhibitor].

**Table I:** List of primers used for RT-qPCR.

Gene	Primer sequence
TNF-α	F: 5′-ATGAGCACAGAAAGCATGATC-3′ R: 5′-TACAGGCTTGTCACTCGAATT-3′
RANTES	F: 5′-TCCAATCTTGCAGTCGTGTTTG-3′ R: 5′-TCTGGGTTGGCACACACTTG-3′
β-actin	F: 5′-GTG GGG CGC CCC AGG CACCA-3′ R: 5′-CTC CTT AAT GTC ACG CAC GAT TTC-3′

TNF-α, tumor necrosis factor-α; RANTES, regulated upon activation, normal T cell expression and secreted. F, forward; R, reverse.

**Table II:** Body and organ weight of the animals (n=60).

Groups	n	BW (g)	PW (g)	LW (g)	SW (g)	KW (g)
0	10	455.9±29.7	1.89±0.27	6.19±0.95	0.93±0.27	3.43±0.91
5	10	437.6±29.4	1.61±0.25	5.91±0.62	1.15±0.33	3.37±0.79
10	10	422.7±28.7^a^	1.43±0.25^a^	5.34±0.81^a^	1.26±0.32	3.44±0.89
15	10	401.3±27.5^a^	1.31±0.26^a^	4.68±0.64^a^	1.17±0.29	3.35±0.88
20	10	392.5±22.8^a^	1.20±0.18^a^	4.15±0.73^a^	1.32±0.41	3.47±1.15
25	10	387.8±26.5^a^	1.07±0.19^a^	3.73±0.71^a^	1.24±0.56	3.51±1.21

BW, body weight; PW, pancreatic weight; LW, liver weight; SW, spleen weight; KW, kidney weight.

a P<0.05 vs. 0 mM/kg/day ethanol (EtOH) + LPS group; denotes a significant difference.

## Abbreviations

ADM: acinar-to-ductal metaplasia
Akt: protein kinase B
CK-19: cytokeratin-19
CP: chronic pancreatitis
ELISA: enzyme-linked immunosorbent assay
GPx: glutathione peroxidase
IKK: inhibitory κB kinase
IL-1: interleukin-1
IL-6: interleukin-6
IL-8: interleukin-8
IRAK: interleukin-1 receptor-associated kinase
IκB: inhibitory κB
JNK: c-Jun amino-terminal kinase
KW: kidney weight
LPS: lipopolysaccharide
LW: liver weight
MAPK: mitogen-activated protein kinase
MDA: malondialdehyde
NF-κB: nuclear factor κB
PanIN: pancreatic intraepithelial neoplasia
PDAC: pancreatic ductal adenocarcinoma
PI3K: phosphatidylinositol-3-kinase
PW: pancreatic weight
RT-qPCR: quantitative reverse transcription-polymerase chain reaction
RANTES: regulated upon activation, normal T cell expression and secreted
SD: Sprague-Dawley rat
siRNA: small-interfering RNA
SOD: superoxide dismutase
SW: spleen weight
TGF-β: tumor growth factor-β
TNF-α: tumor necrosis factor-α
